# Kinetics of Antibody Response in BALB/c and C57BL/6 Mice Bitten by *Phlebotomus papatasi*

**DOI:** 10.1371/journal.pntd.0001719

**Published:** 2012-07-10

**Authors:** Michaela Vlkova, Iva Rohousova, Jitka Hostomska, Lucia Pohankova, Lenka Zidkova, Jan Drahota, Jesus G. Valenzuela, Petr Volf

**Affiliations:** 1 Department of Parasitology, Faculty of Science, Charles University in Prague, Prague, Czech Republic; 2 Vector Molecular Biology Section, Laboratory of Malaria and Vector Research, National Institute of Allergy and Infectious Diseases (NIAID), National Institutes of Health, Rockville, Maryland, United States of America; Institut Pasteur de Tunis, Tunisia

## Abstract

**Background:**

Phlebotomine sand flies are blood-sucking insects transmitting *Leishmania* parasites. In bitten hosts, sand fly saliva elicits specific immune response and the humoral immunity was shown to reflect the intensity of sand fly exposure. Thus, anti-saliva antibodies were suggested as the potential risk marker of *Leishmania* transmission. In this study, we examined the long-term kinetics and persistence of anti-*Phlebotomus papatasi* saliva antibody response in BALB/c and C57BL/6 mice. We also tested the reactivity of mice sera with *P. papatasi* salivary antigens and with the recombinant proteins.

**Methodology/Principal Findings:**

Sera of BALB/c and C57BL/6 mice experimentally bitten by *Phlebotomus papatasi* were tested by ELISA for the presence of anti-saliva IgE, IgG and its subclasses. We detected a significant increase of specific IgG and IgG1 in both mice strains and IgG2b in BALB/c mice that positively correlated with the number of blood-fed *P. papatasi* females. Using western blot and mass spectrometry we identified the major *P. papatasi* antigens as Yellow-related proteins, D7-related proteins, antigen 5-related proteins and SP-15-like proteins. We therefore tested the reactivity of mice sera with four *P. papatasi* recombinant proteins coding for most of these potential antigens (PpSP44, PpSP42, PpSP30, and PpSP28). Each mouse serum reacted with at least one of the recombinant protein tested, although none of the recombinant proteins were recognized by all sera.

**Conclusions:**

Our data confirmed the concept of using anti-sand fly saliva antibodies as a marker of sand fly exposure in *Phlebotomus papatasi*–mice model. As screening of specific antibodies is limited by the availability of salivary gland homogenate, utilization of recombinant proteins in such studies would be beneficial. Our present work demonstrates the feasibility of this implementation. A combination of recombinant salivary proteins is recommended for evaluation of intensity of sand fly exposure in endemic areas and for estimation of risk of *Leishmania* transmission.

## Author Summary

*Leishmania major* is the causative agent of zoonotic cutaneous leishmaniasis and *Phlebotomus papatasi* serve as the major vector. In endemic foci, rodents are the natural reservoirs of this disease. Thus, we studied anti-*P. papatasi* saliva antibody response in BALB/c and C57BL/6 mice that are commonly used as model organisms sensitive and resistant to cutaneous leishmaniasis, respectively. We followed the kinetics and persistence of specific antibody response in both mice strains and we characterized the main *P. papatasi* salivary antigens. We demonstrated that sand fly bites elicit production of specific IgG that reflect the intensity of sand fly exposure. In endemic areas, this could provide useful information about the effectiveness of anti-vector control programs. We also examined the reaction of mice sera with four *P. papatasi* recombinant proteins. Our data indicate that a combination of these proteins could be used instead of crude salivary gland homogenate for the monitoring of anti-sand fly saliva antibodies in natural hosts in endemic foci.

## Introduction

Sand flies (Diptera: Phlebotominae) serve as vectors of leishmaniasis, a neglected disease with symptoms ranging from non-lethal cutaneous to life-threatening visceral form. The causative agents of the disease are protozoan parasites of the genus *Leishmania* which are transmitted to the hosts by the bites of infected sand fly females.

The percentage of infected flies in foci of leishmaniasis fluctuates and humans and animals are more frequently exposed to the bites of uninfected sand flies. Repeated exposure to sand fly saliva elicits anti-saliva antibodies that could be used as a marker of exposure to sand fly bites [1]–[5]. Moreover, the antibodies are sand fly species-specific. Therefore they can be utilized to differentiate between exposure to vector and non-vector species [1], [4], [6]–[9]. In several epidemiological studies, anti-sand fly saliva antibodies were already employed as a reliable tool to monitor exposure to sand fly bites, to evaluate the effectiveness of vector control programs, and in some instances to estimate the risk of *Leishmania* transmission [1], [4], [5], [10]–[14].

In endemic areas sand fly population fluctuate seasonally [15], which may influence host anti-saliva antibody response. However, very little is known about the kinetics and persistence of anti-saliva antibodies in sera of hosts bitten by blood-feeding insects. Few data on antibody kinetics are available from mice, chicken and guinea pigs experimentally exposed to bites of *Triatoma infestans* [16]–[18], from humans bitten by mosquitoes [19]–[22] as well as from humans [4], [23] and dogs [3], [5], [24] bitten by sand flies.

Screening for antibodies is, however, unsuitable for broader use in epidemiological studies until recombinant proteins could be employed instead of the crude salivary gland homogenate, which requires maintenance of sand fly colonies and laboratory dissections of insects. So far, only recombinant salivary proteins from *Lutzomyia longipalpis* have been tested for reactivity with sera of naturally bitten humans, dogs, and foxes [8], [9].

We studied mice antibody response to *P. papatasi*, the main vector of *Leishmania major*, and compared long-term kinetics and persistence of anti-saliva antibodies in BALB/c and C57BL/6 mice that are widely used as model organisms sensitive or resistant to *L. major* infection, respectively. Furthermore, we characterized and compared main *P. papatasi* salivary antigens recognized by sera of experimentally bitten BALB/c and C57BL/6 mice. The reactivity of mice sera was also tested with the four *P. papatasi* recombinant proteins; two Yellow-related proteins (PpSP44/AF335492 and PpSP42/AF335491) and two D7-related proteins (PpSP30/AF335489 and PpSP28/AF335488).

## Methods

### Ethical statement

BALB/c and C57BL/6 mice were maintained and handled in the animal facility of Charles University in Prague in accordance with institutional guidelines and Czech legislation (Act No. 246/1992 coll. on Protection of Animals against Cruelty in present statutes at large), which complies with all relevant European Union and international guidelines for experimental animals. The experiments were approved by the Committee on the Ethics of Animal Experiments of the Charles University in Prague (Permit Number: 24773/2008-10001) and were performed under the Certificate of Competency (Registration Number: CZU 934/05; CZU 307/09) in accordance with the Examination Order approved by Central Commission for Animal Welfare of the Czech Republic.

### Sand flies and salivary gland dissection

A colony of *Phlebotomus papatasi* (originating from Turkey) was reared under standard conditions as described in [25]. Salivary glands were dissected from 4–6-day-old female sand flies, placed into 20 mM Tris buffer with 150 mM NaCl and stored at −20°C.

### Experimental exposure

Twelve mice of BALB/c or C57BL/6 strains (6 weeks old) were divided into experimental and control groups of six mice each. Mice in the experimentally bitten groups were exposed individually to 30 *Phlebotomus papatasi* females (22±0.6 (standard error) blood-fed females per mouse per exposure on BALB/C mice; 26±0.7 (standard error) blood-fed females per mouse per exposure on C57BL/6 mice), once a week in a total of 5 exposures (weeks 1–5). Mice in the control groups remained without any exposure to sand flies. Animals in both groups were anaesthetized (ketamin 150 mg/kg and xylazin 15 mg/kg body weight, intraperitoneally). Blood samples were taken weekly from the tail vein of each mouse one day before exposure to sand flies from week 0 (pre-immune serum) to week 12 and than every other week till the end of the experiment (week 28 for BALB/c mice; week 27 for C57BL/6 mice). In total, mice were followed for 29 and 28 weeks, respectively. Two independent experiments were done for each mice strain.

To test the presence of memory cells, BALB/c mice were additionally exposed to *P. papatasi* bites (21±0.5 (standard error) blood-fed females per mouse) in the week 27.

### Preparation of recombinant proteins

Genes coding for *P. papatasi* salivary gland secreted proteins PpSP28 (AF335488), PpSP30 (AF335489), PpSP42 (AF335491) and PpSP44 (AF335492) were amplified from VR2001-TOPO vector [26] by PCR. Two specific restriction sites (*Nde* I and *Bam* HI) were incorporated into the PCR primers: PpSP28Fw (CATATGAAGTACCCTAGGAATGCCGAT), PpSP28Rev (GGATCCGTACGTTCTTGCGGATTGGTCATC), PpSP30Fw (CATATGCGATTTCCTAGGAATGGAGAC), PpSP30Rev (GGATCCGTATTTCCAAGATTCAATATCAAG), PpSP42Fw (CATATGAAAAGAGATGATGTTGGA), PpSP42Rev (GGATCCCCCTTGACACTTTTCTCC), PpSP44Fw (CATATGAAAAGAGACGATGTTGAA), and PpSP44Rev (GGATCCTTTAGGTTTTCTCACTTC). Afterwards, PCR products were ligated into *E. coli* pGEM-T Easy Vector (Promega) using TA cloning and the ligation products were transformed into *E. coli* competent cells TOP10 (Invitrogen). Vectors were replicated in bacteria and after that, genes restricted by *Nde* I and *Bam* HI enzymes and restricted *E. coli* pET-42 Expression Vectors (Novagen) were ligated. Ligation products were transformed into *E. coli* competent cells TOP10 (Invitrogen) again. Plasmids were isolated from the bacteria, and transformed into *E. coli* BL21 (DE3) gold (Agilent) for expression. *E. coli* lysates were prepared under denaturing conditions and His-tagged proteins were purified by FLPC on a Ni-NTA Superflow column with The QUIaxpressionist kit (Quiagen) according to manufacturers manual.

### Detection of anti-*P. papatasi* saliva antibodies

Anti-*P. papatasi* saliva IgG antibodies and IgG subclasses were measured in sera of BALB/c and C57BL/6 mice using indirect ELISA. Microtiter plate wells were coated with *P. papatasi* salivary gland homogenate (SGH) made by three freeze-thaw cycles (about 60 ng of protein per well). To block free binding sites, washed wells were incubated with 6% low fat dry milk diluted in 20 mM phosphate-buffered saline with 0.05% Tween 20. Mice sera were diluted 1∶200 in 2% low fat dry milk and incubated for 90 min at 37°C for specific IgG or overnight at 4°C for IgG subclasses. Secondary antibodies (goat anti-mouse IgG, IgG1, IgG2a, IgG2b, IgG2c, and IgG3; Serotec) conjugated with horseradish peroxidase (HRP) were diluted and incubated at 37°C as described in Table S1. Orthophenylendiamine and H_2_O_2_ in McIlwein phosphate-citrate buffer (pH 5.5) were used as substrate solution. Absorbance was measured at 492 nm using an Infinite M200 microplate reader (Tecan). The cut-off value was determined as two standard errors of the mean of the absorbance of pre-immune serum. The intensity of booster effect was measured by increased levels of specific antibodies in sera of bitten mice after the last sand fly exposure (comparing week 24 and 28).

Anti-*P. papatasi* IgE were measured in sera of BALB/c mice as described above with the following modifications. Microtiter plate wells were coated with *P. papatasi* SGH (about 300 ng of protein per well). To block the free binding sites, washed wells were incubated with 6% fetal calf serum. Mouse sera were diluted 1∶100 in 2% fetal calf serum. Secondary antibody (rat anti-mouse IgE; BD PharMingen) was diluted and incubated as listed in Table S1.

### Western blot analysis

*Phlebotomus papatasi* SGH (about 10 µg of protein per well) was separated on 10% SDS-PAGE gel under non-reducing conditions using the Mini-Protean III apparatus (BioRad). Salivary proteins were blotted onto a nitrocellulose membrane by Semi-Phor equipment (Hoefer Scientific Instruments) and cut into strips. The strips were then blocked with 5% low fat dry milk in Tris-buffered saline with 0.05% Tween 20 (TBS-Tw) and subsequently incubated with mice sera (week 28 for BALB/c mice; week 5 for C57BL/6 mice) diluted 1∶200 for 1 hour. In the next step the strips were incubated for 1 hour with peroxidase-conjugated goat anti-mouse IgG, IgG1, or IgG2b (Serotec) diluted in TBS-Tw as follows: IgG and IgG1 1∶5000; IgG2b 1∶2000 for BALB/c mice sera and IgG, IgG1 1∶2000 for C57BL/6 mice sera. The chromogenic reaction was developed using a solution containing diaminobenzidine and H_2_O_2_.

Similar protocol was used for western blot analysis with *P. papatasi* recombinant proteins PpSP28, PpSP30, PpSP42, and PpSP44. Briefly, recombinant proteins were loaded on the 10% SDS-PAGE gel (3 µg protein per well) and separated under reducing conditions. BALB/c mice sera (week 28) were diluted 1∶50 and secondary antibody (goat anti-mouse IgG from Serotec) was diluted 1∶1000 in TBS-Tw.

### Mass spectrometry

The proteins from the *P. papatasi* salivary glands used for mass spectrometric analysis were run on the same gel as salivary glands used for western blot analysis. Proteins were visualized by Coomassie Blue G-250 staining (Bio-Rad). The individual bands were cut and incubated with 10 mM dithiothreitol (DTT) and then treated with 55 mM iodoacetamid. Washed and dried bands were digested with trypsin (5 ng, Promega). Alpha-cyano-4-hydroxycinnamic acid was used as a matrix. Samples were measured using a 4800 Plus MALDI TOF/TOF analyzer (AB SCIEX). A peak list from MS spectra was generated by 4000 Series Explorer V 3.5.3 (AB SCIEX) without smoothing. Peaks with local signal to noise ratio greater than 5 were picked and searched by local Mascot v. 2.1 (Matrix Science) against a database of putative salivary protein sequences derived from GenBank. Database search criteria were as follows – enzyme: trypsin, taxonomy: *Phlebotomus*, fixed modification: carbamidomethylation, variable modification: methionine oxidation, peptide mass tolerance: 80 ppm, one missed cleavage allowed. Only hits that scored as significant (p<0.05) are included.

### Statistical analysis

The data obtained by ELISA were subjected to GLM ANOVA and Tukey-Kramer Multiple Comparison procedure to analyze differences in kinetics of anti-*P. papatasi* saliva antibody response between experimentally bitten and control mice at all sampling points. The non-parametric Wilcoxon rank sum test for differences in medians was used for evaluation of booster effect, the comparison of antibody level between week 24 and 28. For correlation tests we used the non-parametric Spearman rank correlation matrix. For all tests statistical significance was regarded as a p-value less than 0.05. All statistical analyses were performed using NCSS 6.0.21 software.

## Results

### Kinetics of anti-*P. papatasi* saliva antibody response in BALB/c mice

To investigate the kinetics and persistence of anti-*P. papatasi* saliva antibody response, experimentally bitten and control mice were followed for 29 weeks. Mice exposed five times to bites of sand flies at one-week interval had significantly increased levels of specific IgG, IgG1, and IgG2b as compared to control group (Figure 1A, C, E). In contrast, specific IgG2a, IgG3, and IgE levels in sera of bitten mice were comparable to non-exposed controls with some differences only at the last data points (Figure S1). No anti-saliva antibodies were detected in any pre-immune sera tested.

**Figure 1:** Anti-sand fly saliva antibody response in BALB/c and C57BL/6 mice bitten by *Phlebotomus papatasi*. BALB/c mice (A, C, E) and C57BL/6 mice (B, D, F) were divided into control (squares) and experimentally bitten groups (circles). Mice in the latter group were exposed to sand fly bites (arrows) in weeks 1–5 and additionally in the week 27 (only BALB/c mice). Levels of specific IgG (A, B); IgG1 (C, D); and IgG2b (E, F) were measured by ELISA at all sampling points. Full circles represent significant difference between control and bitten mice (p<0.05). Data are presented as the means ± standard errors of the means. Two independent studies were done. OD = optical density.

In bitten mice, anti-*P. papatasi* saliva IgG and IgG1 levels increased significantly (p<0.05) after the fourth exposure (Figure 1A, C). IgG2b levels differed between experimental and control group from week 9 onward, with the exception of weeks 10 and 11 (Figure 1E). Anti-saliva IgG increased steadily till the end of the study, while specific IgG2b increased slowly until week 22 followed by a slight decrease at week 24. Anti-saliva IgG1 increased steadily and peaked at week 7 and persisted on this level until the end of the study.

To test the presence of putative memory cells to *P. papatasi* salivary proteins, BALB/c mice were additionally exposed to sand flies 22 weeks after the last exposure (week 27). One week after the booster (at week 28) anti-*P. papatasi* saliva antibodies increased significantly in IgG by 43%, in IgG1 by 80% and in IgG2b by 79% (Figure 1A, C, E).

Positive correlation was found between the number of blood-fed sand fly females during the individual immunization weeks (sum of the blood-fed females from the relevant week and the weeks before) and the corresponding levels of anti-*P. papatasi* IgG (r = 0.62, p<0.0001), IgG1 (r = 0.74, p<0.0001), and IgG2b (r = 0.29, p<0.05) (Figure 2A, C, E). Furthermore, positive correlation was detected between the total amount of blood-fed females and the levels of specific IgG (r = 0.72, p<0.0001) and IgG1 (r = 0.8, p<0.0001) after the fifth sand fly exposure (week 5).

**Figure 2:** Correlation between the intensity of sand fly exposure and the anti-*Phlebotomus papatasi* saliva antibodies. The correlation between the number of blood-fed sand fly females and the levels of anti-saliva antibodies in experimentally bitten BALB/c (A, C, E) and C57BL/6 (B, D) mice was performed using Spearman Rank Correlation Matrix. Positive correlation was detected in specific IgG (A); IgG1 (C); and IgG2b (E) in BALB/c mice and in specific IgG (B); and IgG1 (D) in C57BL/6 mice. OD = optical density.

### Kinetics of anti-*P. papatasi* saliva antibody response in C57BL/6 mice

Experimentally bitten and control mice of C57BL/6 strain were followed in experiments lasting 28 weeks. Five exposures at one-week interval significantly increased levels of specific IgG and IgG1 in bitten mice (Figure 1B, D). In contrast, specific IgG2b, IgG2c, and IgG3 levels of bitten mice were comparable to controls. No anti-saliva antibodies were detected in any pre-immune sera tested.

Similarly to BALB/c mice, anti-*P. papatasi* IgG and IgG1 levels differed significantly between experimentally bitten and control C57BL/6 mice from week 4 onward (Figure 1B, D). Anti-saliva IgG gradually increased until week 8 and then with a slight fluctuation of antibody levels decreased until the end of the study. Specific IgG1 developed with similar kinetics to IgG, however, it peaked earlier (at week 6) and then slowly decreased till the end of the study. Anti-saliva IgG2b, IgG2c, and IgG3 antibodies did not differ between the exposed and control group throughout the study (Figure 1F; Figure S1B, D) with the exception of week 21 for IgG3 subclass (Figure S1D).

We also detected a positive correlation between the number of blood-fed sand fly females during the individual immunization weeks (sum of the blood-fed females from the relevant week and the weeks before) and the corresponding levels of anti-*P. papatasi* IgG (r = 0.80, p<0.0001) and IgG1 (r = 0.86, p<0.0001) (Figure 2B, D). Moreover, positive correlation was detected between the total amount of blood-fed females and the levels of specific IgG (r = 0.85, p<0.0001), IgG1 (r = 0.86, p<0.0001), and IgG2c (r = 0.5, p<0.05) after the fifth sand fly exposure (week 5).

### Identification and characterization of *P. papatasi* salivary antigens

*Phlebotomus papatasi* salivary antigens were studied using sera of experimentally bitten BALB/c and C57BL/6 mice. Only the antibody classes and subclasses shown to be produced in high titers by ELISA were tested in a western blot; specific anti-*P. papatasi* IgG and IgG1 in both mice strains and additionally specific IgG2b in BALB/c mice.

BALB/c mice sera recognized up to 10 protein bands with approximate molecular weights of 70, 65, 51, 49, 47, 35, 31, 30, 23, and 15 kDa, the last three being the most intensively recognized by all BALB/c sera in all IgG subclasses tested. Sera of C57BL/6 mice reacted additionally with the 53 kDa protein but did not recognize the 49 and 47 kDa protein bands. The most intensive reaction in all C57BL/6 mice was detected with the 65, 53, and 30 kDa protein bands in IgG as well as in IgG1 (Figure 3). Comparison of two mice strains therefore revealed an interesting difference in recognition of four protein bands of 53, 51, 49, and 47 kDa. No reaction was detected with any pre-immune mice sera tested (Figure 3).

**Figure 3:** Anti-sand fly saliva antibody response in BALB/c and C57BL/6 mice experimentally bitten by *Phlebotomus papatasi*. (A) Total protein profile, Coomassie blue-stained SDS-PAGE gel with *P. papatasi* salivary gland homogenate. (B) Western blot of *P. papatasi* salivary proteins recognized by IgG, IgG1, or IgG2b from sera of *P. papatasi*-bitten BALB/c (week 28) and C57BL/6 mice (week 5). Pre-immune sera of BALB/c and C57BL/6 mice were used as negative controls (Neg).

In BALB/c mice, the 51 kDa protein was recognized only by one out of 5 sera tested in IgG and IgG1, while in C57BL/6 mice, this protein band was recognized by all mice sera tested in IgG1 and by two out of five sera tested in IgG. Anti-*P. papatasi* IgG2b antibodies reacted consistently with the 65, 35, 31, 30, 23, and 15 kDa proteins (Figure 3).

In C57BL/6 mice, 70, 65, 53, 31, and 30 kDa proteins were recognized by all mice sera tested (IgG as well as IgG1), while the 51, 35, 23, and 15 kDa antigens were recognized by some sera only (Figure 3). Specific IgG1 of C57BL/6 mice predominantly recognized the 65, 53, 51, 31, and 30 kDa antigens (Figure 3).

Mass spectrometry analysis identified the salivary proteins with the same mobility in the SDS-PAGE as the proteins recognized by the sera of experimentally bitten mice as the Yellow-related proteins (GenBank acc. no. AF335492 and AF335491), apyrase (AF261768), D7-related proteins (AF335489; AF335488), antigen-5 protein (DQ205724), and proteins of the SP15 protein family (AY628879, AY628880; AF335486; AF335485) (Table 1).

**Table 1:** *Phlebotomus papatasi* salivary proteins recognized by sera of bitten mice.

MW	NCBI acc.number	Best match to NR protein database		
(kDa)		Sequence name	E-value	Protein family
70	N.D.	N.D.	N.D.	N.D.
65	N.D.	N.D.	N.D.	N.D.
53	N.D.	N.D.	N.D.	N.D.
51	AF335492	44 kDa yellow-related salivary protein (PpSP44)	0.00E+00	yellow-related
49	N.D.	N.D.	N.D.	N.D.
47	AF335491	42 kDa yellow-related salivary protein (PpSP42)	0.00E+00	yellow-related
35	AF261768	salivary apyrase (PpSP36)	0.00E+00	apyrase
31	AF335490	32 kDa salivary protein (PpSP32)	1.10E−05	PpSP32-like
30	AF335489	30 kDa D7-related salivary protein (PpSP30)	4.50E−12	D7-related
30	DQ205724	29 kDa antigen 5-related salivary protein	7.10E−05	antigen 5-related
23	AF335488	28 kDa D7-related salivary protein (PpSP28)	0.00E+00	D7-related
15	AY628879	SP-15 protein	1.80E−05	PpSP15-like
15	AY628880	SP-15 protein	3.50E−07	PpSP15-like
15	AF335486	14 kDa salivary protein (PpSP14)	0.00E+00	PpSP15-like
15	AF335485	12 kDa salivary protein (PpSP12)	0.00E+00	PpSP15-like

N.D. – not determined.

### Reactivity of anti-saliva antibodies with the *P. papatasi* recombinant proteins

The reactivity of PpSP44 (yellow related protein), PpSP42 (yellow related protein), PpSP30 (D7 related protein), and PpSP28 (D7 related protein) recombinant proteins was studied using sera from BALB/c mice exposed to *P. papatasi* bites and positive for anti-*P. papatasi* IgG antibodies. Sera of control mice did not recognize any of the recombinant proteins tested. The most intensive reaction was detected with the PpSP30, although, this protein was not recognized by all sera tested (4 out of 5). Three out of five mice sera reacted with the PpSP42 and PpSP44 recombinant proteins and very weak reaction was detected with the PpSP28 recombinant protein in two out of five mice sera (Figure 4).

**Figure 4:** Reactivity of anti-*Phlebotomus papatasi* saliva IgG with *P. papatasi* recombinant proteins. Sera from BALB/c mice experimentally bitten by *P. papatasi* (Bitten mice) that were positive for anti-*P. papatasi* IgG (OD>cut-off: 0.19) were tested by Western blot analysis against (A) *P. papatasi* salivary gland homogenate, (B) a combination of bacterially-expressed PpSP42 and PpSP28 (Yellow-related protein AF335491 and D7-related protein AF335488, respectively), and (C) a combination of bacterially-expressed PpSP44 and PpSP30 (Yellow-related protein AF335492 and D7-related protein AF335489, respectively). The SDS-PAGE protein profiles of the *P. papatasi* salivary gland homogenate as well as the recombinant proteins were blotted and stained by Amido Black. Pre-immune sera of BALB/c mice were used as the controls (Neg).

## Discussion

This study describes in detail long-term kinetics and persistence of anti-*P. papatasi* saliva antibodies in sand fly-exposed BALB/c and C57BL/6 mice strains that are widely used as model organisms sensitive or resistant to *Leishmania* infection, respectively (e.g. [27], [28]).

Four IgG subtypes have been described in mice: IgG1, IgG2a, IgG2b, and IgG3. Additionally, certain strains such as C57BL/6 produce the IgG2c subclass instead of IgG2a [29]. The nomenclature of murine IgG subtypes does not correlate with the subtypes of human or canine IgG. The most abundant subclass is IgG1; it binds to Fc-receptors of mast cells and basophils, and it mediates the immediate hypersensitivity reactions. Both IgG1 and IgG2a activate the complement cascade via the alternative pathway, whereas IgG2b employs the classical pathway of complement activation [30]. Moreover, production of IgG1 is the marker of Th2 profile of immune response in mice, while IgG2a predicts Th1 type of immune response in these animals [31].

We showed that repeated exposure to sand fly bites elicits increased levels of anti-saliva IgG and IgG1 in both BALB/c and C57BL/6 strains, and additionally IgG2b in BALB/c mice. In comparison, higher levels of specific IgG were detected in BALB/c mice. This finding complies well with the fact that BALB/c mice mostly respond to repeating antigens by Th2 humoral immune response while C57BL/6 mice produce mainly Th1 cellular response [30]. It seems that *P. papatasi* saliva elicits mainly production of specific IgG1 subclass, which suggests the polarization to the Th2 type of immune response in bitten mice regardless of the strain. The production of anti-sand fly saliva IgG1 was previously described in BALB/c mice repeatedly bitten by *Lutzomyia longipalpis*, but they did not observe any production of neither IgG2a nor IgG2b [32]. As the composition of sand fly saliva varies in different sand fly species [33] and the sand fly saliva compounds elicit different profile of specific antibody response [34], this could be the feasible explanation for the production of different antibody subclasses in mice bitten by different sand fly species. To our knowledge, there are no data available about the anti-sand fly saliva antibody subclasses elicited by sand fly feeding in the C57BL/6 mice. In Swiss Webster mice immunization by *P. ariasi* saliva produced also predominantly IgG1 antibodies [34]. Production of specific IgG2b in BALB/c mice compared to the absence of this antibody subclass in C57BL/6 mice may be the result of different cytokine responses in both mice strains against sand fly saliva. The switch to IgG2b subclass is initialized by production of TGF-β [35], a suppressive cytokine that blocks the activation of lymphocytes and monocytes derived phagocytes. This could positively contribute to the susceptibility of BALB/c mice to *Leishmania* parasites.

Importantly, positive correlation was found in both mice strains between the intensity of sand fly exposure and the levels of specific antibodies in aforementioned subclasses. Our results correspond well to previously published data showing that the antibody response in dogs [3], [5] as well as in humans [4] reflected the intensity and the time-course of sand fly exposure.

We found that sand fly exposure did not affect the production of IgG2a and IgG3 in BALB/c mice, and IgG2b, IgG2c, and IgG3 in C57BL/6 mice. Neither did the levels of specific IgE differ significantly between non-exposed and exposed groups of mice, and the IgE kinetics showed high variation during the study. Similarly, high fluctuation in specific IgE response was detected in humans [11], [23] and dogs [3] bitten by *Lutzomyia longipalpis* in the field as well as under laboratory conditions. While some of the individuals and animals presented high levels of specific IgE, others did not mount specific IgE response at all [3], [11], [23].

To mimic the situation commonly occurring in endemic foci of leishmaniases, where sand fly-free periods last up to 6 months [15], BALB/c mice were exposed to *P. papatasi* bites again 23 weeks after the last sand fly exposure. This single sand fly exposure elicited statistically significant increase of anti-*P. papatasi* IgG, IgG1, IgG2b which suggests the persistence of memory cells generated during the previous round of exposures. This could be related to the “previous sand fly season” in the field. Furthermore, in both mice strains, the differences between non-exposed and exposed groups of mice in production of specific IgG1 and IgG2b were detectable from week four or nine, respectively, until the end of the study. Similarly, the levels of specific IgG, IgG1, and IgG2 in sera of dogs exposed to *L. longipalpis* or *P. perniciosus* bites differed significantly from pre-immune sera for more than 14 weeks after the last sand fly exposure [3], [5]. In individuals repeatedly bitten by *P. argentipes*, elevated levels of specific antibodies persisted after the 30-day sand fly-free period, although anti-saliva antibodies significantly decreased throughout this time [4]. Thus, regardless the host-sand fly combination, anti-sand fly saliva antibodies can persist in sera of repeatedly bitten hosts until the next sand fly season.

We also characterized the reactivity of mice sera with *P. papatasi* salivary proteins as well as with selected recombinant proteins. Mice sera of BALB/c and C57BL/6 strains reacted with up to eleven *P. papatasi* antigenic protein bands. The 30 kDa protein band recognized by both mice strains was identified by mass spectrometry as a mixture of a D7-related (AF335489) and an antigen 5-related (DQ205724) protein. The other proteins which were intensively recognized either by BALB/c (47, 23, and 15 kDa proteins) or by C57BL/6 mice (65, 53, and 51 kDa proteins) were determined as members of the Yellow-related protein family (51 kDa - AF335492, 47 kDa - AF335491), D7-related protein family (23 kDa – AF335488), and SP-15 protein family (15 kDa – AY628879, AY628880, AF335486, AF335485). The 70, 65, 53, and 49 kDa bands were not identified by mass spectrometry. Our results correspond to previously published data, where the human and BALB/c mice IgG antibodies recognized preferentially the *P. papatasi* 30 kDa protein band [1], [14].

To our knowledge, the only study describing the reactivity of specific IgG subclasses with *P. papatasi* antigens was performed on humans [14]. In accordance with our results, the 30 kDa D7-related protein was also found to be the most immunogenic antigen in all human antibody subclasses tested [14]. Taken together, our data complies well with previously published studies, where Yellow-related proteins, D7-related proteins, as well as SP-15 proteins from *P. papatasi* saliva were identified as potent antigens for mice and humans [1], [14].

Sera of BALB/c mice experimentally bitten by *P. papatasi* were tested also with four bacterially expressed recombinant proteins belonging to two salivary protein families: Yellow-related proteins (PpSP44/AF335492 and PpSP42/AF335491) and D7-related proteins (PpSP30/AF335489 and PpSP28/AF335488). Within the salivary gland homogenate, sera reacted with proteins identified as PpSP42, PpSP30, and PpSP28 proteins, but no reaction was detected with PpSP44. In contrast, PpSP30 and PpSP44 recombinant proteins were strongly recognized and PpSP42 gave a weak reaction. Reaction of anti-saliva IgG with recombinant proteins may, however, differ between mouse strains. For example, the C57BL/6 mice reacted predominantly with PpSP42 and PpSP28 recombinant proteins (data not shown). Although none of the recombinant proteins were recognized by all sera. Each mouse serum tested reacted with at least one of the recombinant proteins.

Our data suggest that recombinant proteins could be used as markers of sand fly exposure instead of crude salivary gland homogenates, ideally as a mixture of several different proteins to cope with various host species and individual reactivity of each serum sample. In sand flies this concept has been demonstrated using *Lutzomyia longipalpis* recombinant proteins; the reactivity of anti-*L. longipalpis* seropositive human sera with the salivary gland sonicate was comparable to the reaction with the combination of the two *L. longipalpis* recombinant Yellow-related proteins (LJM11/AY445935 and LJM17/AF132518) [8].

In conclusion, we detected a significant increase of specific IgG and IgG1 in exposed mice of both strains, and of IgG2b in exposed BALB/c mice. The other IgG subclasses were comparable to controls. Specific IgG response was shown to reflect the intensity of sand fly exposure and furthermore, anti-*P. papatasi* saliva antibody response persisted in mice for more than 5 months. Thus, in endemic areas the antibodies could persist till the following sand fly season. The 30 kDa band recognized by sera of experimentally bitten BALB/c as well as C57BL/6 mice was identified as a mixture of D7-related and antigen 5-related proteins. Moreover, the reactivity of mice sera with PpSP44, PpSP42, PpSP30, and PpSP28 recombinant proteins suggested that their combination could substitute the salivary gland homogenate. Taken together, the kinetics, persistence and the individual variability of anti-sand fly saliva antibody response are important aspects to consider in further experiments, where anti-saliva antibodies are used as the markers of sand fly exposure.

## Supporting Information

Figure S1 **Anti-sand fly saliva antibody response in BALB/c and C57BL/6 mice bitten by** ***Phlebotomus papatasi*** **.** BALB/c mice and C57BL/6 mice were divided into control (squares) and experimentally bitten groups (circles). Mice in the latter group were exposed to sand fly bites (arrows) (30 *P. papatasi* females per week) in weeks 1–5 and additionally in the week 27 (only BALB/c mice). Anti-*P. papatasi* saliva antibodies - IgG2a (A), IgG3 (C), and IgE (E) in BALB/c mice and IgG2c (B) and IgG3 (D) in C57BL/6 mice - were measured using ELISA as described in Methods. Data are presented as the means ± standard errors of the means. Two independent studies were done. OD = optical density.
(TIF)

Table S1 **Dilution and incubation time of secondary antibodies.**
(DOC)
